The article "Dexmedetomidine Attenuates LPS-Induced Acute Lung Injury in Rats by Activating the Nrf2/ARE Pathway" was retracted in 2023. Reasons: signs of a paper mill; suspected computer-generated content; unreliable results or conclusions; concerns about the data.

# Dexmedetomidine Attenuates LPS-Induced Acute Lung Injury in Rats by Activating the Nrf2/ARE Pathway

**DOI:** 10.1155/2022/4185195

**Published:** 2022-04-11

**Authors:** Yuandong Qiu, Zhiwei Tang

**Affiliations:** ^1^Department of Anesthesiology, Koiqeung Memorial Hospital, Guangzhou, Guangdong, China; ^2^The Fifth Affiliated Hospital of Southern Medical University, Guangzhou, Guangdong 510900, China

## Abstract

**Background:**

To investigate the effect of dexmedetomidine (Dex) on lipopolysaccharide (LPS)-induced acute lung injury (ALI) in rats and its mechanism.

**Methods:**

Eighteen SD rats were randomly divided into 3 groups (6 rats in each group): control group (intratracheal instillation of saline), ALI group (intratracheal instillation of 5 mg/kg LPS), and ALI-Dex group (tail vein injection of 50 *μ*g/kg/h Dex + intratracheal instillation of LPS). Subsequently, the water content of lung tissues was assessed using the wet-dry (W/D) ratio and the histopathological changes of lung tissues using H&E staining. Further activities of ROS, SOD, and GSH-Px in lung tissues of rats were measured by an automatic biochemistry analyzer. ELISA was performed to detect TNF-*α*, IL-1*β*, and IL-6 expression in alveolar lavage fluid (BALF) and Western blot to detect the expression of Nrf2/ARE pathway-related proteins.

**Results:**

After Dex treatment, a reduction in water content in lung tissue and an improvement of lung injury were found in the ALI rats. Compared with the ALI group, rats in the ALI-Dex group had decreased ROS activity and increased activities of SOD and GSH-Px in lung tissues. Dex-treated rats were also associated with a decrease in TNF-*α*, IL-1*β*, and IL-6 expression in alveolar lavage fluid (BALF). Additionally, increased expression levels of HO-1 and NQO1 in lung tissues and elevated expression of Nrf2 in the nucleus were shown in the ALI-Dex group compared with the ALI group.

**Conclusion:**

Dex alleviates LPS-induced ALI by activating the Nrf2/ARE signaling pathway.

## 1. Introduction

Acute lung injury (ALI) and acute respiratory distress syndrome (ARDS) are common and severe complications in critically ill patients and are prevalent in intensive care units [1]. ARDS affects at least 10% of patients in the intensive care unit, with a mortality rate of about 40% [2]. ALI is an acute inflammatory disease caused by disruption of the pulmonary endothelial and epithelial barriers [3]. Its pathological features include loss of alveolar-capillary membrane integrity, uncontrolled migration of neutrophils, and uncontrolled release of proinflammatory factors [4]. Given the pathogenesis, most clinical treatments are aimed at improving the respiratory status of patients, such as using 3-hydroxy-3-methylglutaryl coenzyme A (HMG-CoA) reductase inhibitors (statins) and *β*-2 agonists. In addition, glucocorticoids have been reported to accelerate the regression of alveolar edema by reducing inflammation and upregulating alveolar to transport salt and water [5]. Despite encouraging early preclinical evidence for these drugs, phase III clinical trials have shown unsatisfactory results [6]. To date, significant advances have been made in the treatment strategies of ALI and understanding of related respiratory physiology, but the annual mortality rate of ALI remains at 40%. Therefore, the search for new drugs and the development of appropriate therapeutic strategies are of great urgency.

The article "Dexmedetomidine Attenuates LPS-Induced Acute Lung Injury in Rats by Activating the Nrf2/ARE Pathway" was retracted in 2023. Reasons: signs of a paper mill; suspected computer-generated content; unreliable results or conclusions; concerns about the data.

Dexmedetomidine (Dex) is a highly effective and selective alpha-2 adrenergic receptor agonist with sedative and analgesic properties. It is widely used in the anesthesia of critically ill patients and can also improve amnesia and sympathetic nervous system [7]. Further studies on the function of Dex have found that Dex can improve postoperative recovery in a variety of diseases [8]. Dex can reduce mortality as well as ventilator use in patients with sepsis [9]. Dex can decrease the levels of inflammatory mediators (e.g., cytokines and interleukins) and immunosuppression, thus improving the prognosis of the systemic inflammatory response syndrome that is often triggered by surgical resection of tumors [9, 10]. In addition, Gu et al. found that in ALI induced by renal ischemia-reperfusion, Dex improved pulmonary microvascular hyperpermeability to protect the lung tissue [11]. These studies suggest that Dex, in addition to its highly effective anesthetic effect with low side effects, also has the ability to slow down the development of diseases caused by immune dysregulation. In recent years, it has been found that Dex has a positive effect on lipopolysaccharide (LPS)-induced ALI through the high mobility group protein B1 (HMGB1)-mediated TLR4/NF-*κ*B and PI3K/Akt/mTOR pathways [12]. LPS can combine with the TLR4 group on the surface of cell membrane to transfer the signal to the interior of immune cells. Activate myeloid differentiation factor 88 (MyD88)-dependent signaling pathway and TLR domain adaptor protein (TRIF)-dependent signaling pathway, activate mitogen activated protein kinase (MAPK), and activate NF-*κ*B. To activate the MAPK/NF-*κ*B signal pathway, activated NF-*κ*B enters the nucleus and acts with the promoter of related genes, so as to promote the release of inflammatory factors or chemokines and cause inflammatory response [13]. The Nrf2/ARE signaling pathway has been proved to be one of the mechanisms of ALI or ARDS [14]. However, there is no study on the mechanism that Dex regulates ALI through the Nrf2/ARE signaling pathway. Therefore, in this study, we attempt to elucidate the effect of Dex on LPS-induced ALI and its mechanism by constructing an ALI rat model.

The article "Dexmedetomidine Attenuates LPS-Induced Acute Lung Injury in Rats by Activating the Nrf2/ARE Pathway" was retracted in 2023. Reasons: signs of a paper mill; suspected computer-generated content; unreliable results or conclusions; concerns about the data.

## 2. Materials and Methods

### 2.1. Construction of Rat Models of Acute Lung Injury

Eighteen male SD rats of 6–8 weeks of age, weighing 180 g–220 g, were randomly divided into three groups (6 rats in each group): control group, ALI group, and ALI-Dex group. The ALI group received intratracheal instillation of 8 mg/kg LPS [12]. The ALI-Dex group was first given tail vein injection of 50 *μ*g/kg/h Dex for 90 min (50 *μ*g/kg/h, total dose ≤75 *μ*g/kg), and 30 min after the injection, received the same procedure as the ALI group. The control group had intratracheal instillation of an equal volume of saline. All rats were killed 6 h after LPS induction to obtain lung tissues and alveolar lavage fluid (BALF) and store them at −80°C. Lung tissues for H&E staining were fixed and stored in 4% paraformaldehyde. All research protocols involving animals in this study after adaptive feeding were approved by the Institutional Animal Ethics Committee of the Guangdong Provincial Medical Laboratory Animal Center (C202201-2) and carried out according to the approved guidelines.

### 2.2. Lung Wet-to-Dry Weight (W/D) Ratio

The water content of rat lung tissue was measured by wet/dry (W/D) ratio. The right lung tissue was separated from the obtained rat lungs and weighed; the result was recorded as wet weight. Then, the lung tissue was placed in a constant temperature incubator at 80°C for more than 48 h until the weight no longer changed; this weight was the dry weight. Finally, the W/D ratio was calculated.

### 2.3. H&E Staining

Lung tissues of the same site of rats in each group were perfused with 4% paraformaldehyde and then fixed with 4% paraformaldehyde for another 12 h. After fixation, the tissue samples were embedded in paraffin and sectioned (5 *μ*m). The sections were rinsed 3 times with PBS and stained with hematoxylin at room temperature for 5 min, followed by differentiation using hydrochloric acid alcohol and bluing with 1% v/v ammonia. Subsequently, the samples were stained with eosin for 30 s after rinsing with tap water. Finally, the sections were dehydrated with alcohol, treated with xylene, and sealed. The histopathological changes in the lung tissues were observed under an inverted microscope.

### 2.4. ROS, SOD, and GSH-Px Activities in Lung Tissue

First, 50 mg of lung tissue from each group was collected and placed in a homogenization tube, followed by addition of 1 mL of precooled PBS buffer into the tube. Then, a low-temperature homogenizer was used to break down the tissues. The cell suspension was collected, centrifuged, and the supernatant was transferred to a new centrifuge tube. The activities of ROS, SOD, and GSH-Px in the lung tissues of each group were measured by an automatic biochemistry analyzer (Olympus, Japan).

The article "Dexmedetomidine Attenuates LPS-Induced Acute Lung Injury in Rats by Activating the Nrf2/ARE Pathway" was retracted in 2023. Reasons: signs of a paper mill; suspected computer-generated content; unreliable results or conclusions; concerns about the data.

### 2.5. ELISA Assay

After 6 h of LPS or saline administration, the lungs were lavaged 3 times with 500 *μ*l of sterile PBS (total volume 1.5 ml) to collect BALF. Then, 1 mL of BALF was taken from each group in a 1.5 mL centrifuge tube and centrifuged at 4°C and 12000 g for 10 min. The cell debris was removed, and the supernatant was collected in a new centrifuge tube. Subsequently, the levels of TNF-*α*, IL-1*β*, and IL-6 in BALF were measured according to the instructions of the ELISA kits (Nanjing Jiancheng Bioengineering Institute, China).

### 2.6. Western Blot

Nrf2 was extracted from the lung tissues using the nuclear protein extraction kit, and HO-1 and NQO1 proteins were extracted using RIPA buffer. The protein concentrations were then determined by BCA protein assay (Thermo Fisher, USA). Equal amounts of proteins were extracted and separated by 10% SDS-PAGE. The target proteins were then transferred to PVDF membranes. The membranes were blocked with 5% skim milk for 1 h and incubated with primary antibodies at 4°C overnight. The next day, the membranes were incubated with the corresponding secondary antibodies at room temperature for 1 h, followed by rinsing step with TBST. The membranes were placed in a gel imaging and analysis system with ECL chemiluminescent substrate, and images were acquired using Image Lab^TM^ software to analyze the grayscale values of the bands. *β*-actin was used as an internal reference for whole-cell proteins, while Lamin B was for nuclear proteins.

### 2.7. Statistics Analysis

SPSS 26.0 software was used for statistical analysis. The experimental data were expressed as mean ± standard deviation (SD). One-way analysis of variance compared the difference between groups. *P* < 0.05 suggested a statistically significant difference.

## 3. Results

### 3.1. Dexmedetomidine Relieves Acute Lung Injury Caused by LPS

The results of the W/D ratio showed that LPS caused a significant increase in the water content of lung tissues, while Dex treatment significantly reduced the water content (Figure 1(a)). H&E staining showed no apparent pathological damage in the control group, with normal alveolar structure and intact alveolar wall. By contrast, in the ALI group, the alveolar structure was destroyed, and the alveolar wall was thickened and edematous. Also, ALI rats had a large number of inflammatory cell infiltrates and erythrocyte exudates observed in the alveolar wall and alveolar cavity. After Dex treatment, the thickening and edema of the alveolar, the inflammatory infiltration, and erythrocyte exudation mentioned in ALI rats were improved (Figure 1(b)).

The article "Dexmedetomidine Attenuates LPS-Induced Acute Lung Injury in Rats by Activating the Nrf2/ARE Pathway" was retracted in 2023. Reasons: signs of a paper mill; suspected computer-generated content; unreliable results or conclusions; concerns about the data.

### 3.2. Dexmedetomidine Attenuates Oxidative Stress in Rats with Acute Lung Injury

The results of biochemical assays of lung tissue lysates showed that LPS-induced ALI and significantly increased ROS content in lung tissues while decreasing SOD and GSH-Px activities. In contrast, the ROS content was decreased and SOD and GSH-Px activities became higher in the lung tissues after Dex treatment (Figures 2(a)–2(c)).

### 3.3. Dexmedetomidine Attenuates Inflammation in Rats with Acute Lung Injury

The ELISA results showed (Figures 3(a)–3(c)) that the levels of inflammatory factors TNF-*α*, IL-1*β*, and IL-6 were significantly higher in the BALF of rats in the ALI group compared with the control group (*P* < 0.05). Their expression levels in BALF, however, were decreased after Dex treatment (*P* < 0.05).

### 3.4. Dexmedetomidine Activates the Nrf2/ARE Pathway in the Lung Tissue of Rats with Acute Lung Injury

Western blot showed (Figures 4(a)–4(d)) that compared with the control group, Nrf2 expression in the nucleus and cellular HO-1 and NQO1 protein expression were significantly lower in the lung tissue in the ALI group (*P* < 0.05). In comparison with the ALI group, the expression of such 3 proteins was all significantly upregulated after Dex treatment (*P* < 0.05).

## 4. Discussion

In this study, we found that in the LPS-induced rat ALI model, DEX could reduce the water content of the lung tissue and improve the alveolar thickening, edema, inflammatory infiltration, and erythrocyte extravasation in ALI rats. After DEX treatment, the activity of ROS in the lung tissue of the rats in the ALI-Dex group decreased, the activities of SOD and GSH-Px increased, and the expressions of TNF-*α*, IL-1*β*, and IL-6 in BALF were also decreased. This indicates that DEX can attenuate oxidative stress and inflammatory response in ALI rats. In addition, compared with the ALI group, the expression levels of HO-1 and NQO1 in the lung tissue of the ALI-Dex group increased, and the expression of Nrf2 in the nucleus increased, indicating DEX able to activate the Nrf2/ARE pathway.

ALI is a progressive and destructive disease. Various direct and indirect factors result in lung injury and subsequent ALI, with endotoxemia being a common causation [15]. It is reported that systemic diseases caused by various pathogenic factors inside and outside the lung are the root causes of pediatric ALI/ARDS. In addition, the incidence rate of ALI/ARDS in sepsis patients is 25–50%, causing serious complications and death [16, 17]. Moreover, a large number of clinical transfusions, multiple trauma, and aspiration can also lead to ALI/ARDS, with an incidence rate of 40%, 11–25%, and 9%, respectively [18, 19]. Although a variety of drug options have been developed for ALI, treating the primary affection is the first principle in the treatment of ALI because ALI is only a terminal pathological process of many conditions. The promising efficacy of Dex has been demonstrated in the treatment of multiple diseases. This highly selective *α*2-adrenergic receptor inhibitor with anti-inflammatory effects is often used as a sedative for critically ill patients [20]. Sun et al. showed that Dex could protect glial cells by reducing apoptosis and protecting neurons, thus preserving brain function and ultimately improving the prognosis of sepsis [21]. Zheng et al. found that Dex reduced HIF-1alpha expression and upregulated miR-155 expression in ovarian cancer cells, thereby inhibiting cell proliferation, migration, and invasion and promoting apoptosis [22]. Kong et al. reported that Dex attenuated LPS-induced myocardial injury in mice with septic cardiomyopathy, suggesting that Dex has some protective functions against LPS [23]. According to the results of our study, Dex can effectively alleviate LPS-caused ALI. This means that the clinical use of Dex has been extended.

The article "Dexmedetomidine Attenuates LPS-Induced Acute Lung Injury in Rats by Activating the Nrf2/ARE Pathway" was retracted in 2023. Reasons: signs of a paper mill; suspected computer-generated content; unreliable results or conclusions; concerns about the data.

Many studies have also pointed out that Dex can inhibit body damage caused by excessive oxidative stress. Chen et al. found that Dex reduced oxidative stress and apoptosis by inhibiting the ROS/JNK pathway, preventing acute stress kidney injury in rats [24]. Cai et al. revealed that Dex downregulated PKC-*α* to inhibit the NOX2/ROS signaling pathway, decreased VLA-4 and LFA-1 expression, and ultimately led to a decrease in monocyte-endothelial adherence [25]. In our study, we found that after DEX treatment, the concentrations of TNF-*α*, IL-1*β*, and IL-6 in the BALF of rats were decreased, the activity of ROS in the lung tissue was decreased, and the activities of SOD and GSH-Px were increased. These findings suggest that Dex can counteract dysregulated oxidative stress in the organism, and we got consistent results that Dex attenuates oxidative stress and excessive inflammatory response in ALI rats. It is known that dysregulation of inflammatory response and oxidative stress is a crucial factor leading to ALI. Thus, it can be concluded that mechanistically, Dex attenuates LPS-caused ALI by regulating the inflammatory response and oxidative stress.

The Nrf2/ARE pathway plays a critical role in developing many diseases and is essential for natural antioxidant regulation in cells. Many antioxidant drugs function through the Nrf2/ARE pathway. Nrf2, once activated, binds to endogenous antioxidant response elements (AREs) and enables the expression of many antioxidant genes and proteins to maintain cellular redox homeostasis and normal metabolism [26]. Conversely, dysregulation of the Nrf2/ARE pathway can develop many inflammatory diseases, including cancer, Alzheimer's disease, Parkinson's disease, and diabetes [27]. Therefore, this signaling pathway is considered a regulator of oxidative stress and inflammatory diseases and conditions. Some Nrf2/ARE inducers, such as bardoxolone, dimethyl fumarate, and sulforaphane, have entered phase III clinical trials [28] and have been used as chemopreventive agents for cancer, diabetes, neurological diseases, or as therapeutic agents for inflammation-related diseases, showing good progress [29]. It has also been shown that Nrf2, which is mainly expressed in epithelium and alveolar macrophages, protects the lung from oxidative stress, alveolar apoptosis, extracellular matrix protein hydrolysis, and chronic inflammation [30]. Activated Nrf2 has a therapeutic role in idiopathic pulmonary fibrosis, asthma, bronchopulmonary dysplasia, ALI, and other diseases [31]. Nrf2 translocation into the nucleus contributes to activating ARE-dependent expression of genes and proteins involved in antioxidant defence and cytoprotecting [32]. The Nrf2/ARE signaling pathway is important in preventing the occurrence of ALI/ARDS, and activation of Nrf2 can prevent or reduce the severity of ALI/ARDS [33]. Furthermore, activated Nrf2 was translocated into the nucleus to regulate the expression of HO-1-related genes. Activated HO-1 inhibits the inflammatory cascade and reduces inflammation-induced ALI, thereby protecting organs [34]. Dex, in our study, significantly increased Nrf2 aggregation in the nucleus, suggesting that Dex treats ALI through the Nrf2/ARE pathway. Compared with the above three Nrf2/ARE inducers, bardoxolone, dimethyl fumarate, and lycopene, Dex is already a pharmacokinetic Nrf2/ARE pathway activator approved by drug administrations and can be considered for all diseases and conditions related to the blocked Nrf2/ARE pathway. This study provides a theoretical basis for the development of new anti-inflammatory drugs and provides guidance for the clinical application of DEX as anti-inflammatory drugs.

The article "Dexmedetomidine Attenuates LPS-Induced Acute Lung Injury in Rats by Activating the Nrf2/ARE Pathway" was retracted in 2023. Reasons: signs of a paper mill; suspected computer-generated content; unreliable results or conclusions; concerns about the data.

## 5. Conclusion

In summary, Dex reduces oxidative stress and inflammatory responses by activating the Nrf2/ARE signaling pathway, thus ultimately alleviating LPS-induced ALI. Our results suggest that Dex has the potential to clinically treat LPS-induced ALI. However, our study has no further Nrf2/ARE blockade assay to verify the specificity of the Nrf2/ARE pathway in the antioxidant and anti-inflammatory effects of Dex. The way of activation of the Nrf2/ARE pathway by Dex also requires further exploration to provide a more comprehensive theoretical basis for the following clinical trials.

## Figures and Tables

**Figure 1:** Dexmedetomidine alleviates acute lung injury caused by LPS. (a) Wet-to-dry ratio for assessing the water content of lung tissues. (b) H&E staining to observe the pathological changes of lung tissues. *N* = 6.  ^*∗*^ ^*∗*^*P* < 0.01 vs. the control group; ^##^*P* < 0.01 vs. the ALI group.

**Figure 2:** Dexmedetomidine attenuates oxidative stress in rats with acute lung injury. The ROS (a) content and SOD (b) and GSH-Px activities (c) in the lung tissue of rats measured by an automatic biochemistry analyzer. *N* = 6.  ^*∗*^ ^*∗*^*P* < 0.01 vs. the control group; ^##^*P* < 0.01 vs. the ALI group.

**Figure 3:** Dexmedetomidine attenuates the inflammatory response in rats with acute lung injury. ELISA for TNF-*α* (a), IL-1*β* (b), and IL-6 (c) in alveolar lavage fluid of rats. *N* = 6,  ^*∗*^ ^*∗*^*P* < 0.01 vs. the control group; ^##^*P* < 0.011 vs. the ALI group.

**Figure 4:** Dexmedetomidine activates the Nrf2/ARE pathway in the lung tissue of rats with acute lung injury. Western blot detection of nucleus Nrf2 (a) and the grayscale analysis (b). Western blot detection of cellular HO-1, NQO1 (c), and the grayscale analysis (d).  ^*∗*^ ^*∗*^*P* < 0.01 vs. the control group; ^##^*P* < 0.01 vs. the ALI group.

## Data Availability

The data used to support the findings of this study are available from the corresponding author upon request.
